# A2/B1 Promotes NRF2 mRNA Stability and Inhibits Ferroptosis and Cell Proliferation in Breast Cancer Cells

This article has been retracted.

**DOI:** 10.1155/2023/2620738

**Published:** 2023-04-14

**Authors:** Yan Huang, Jingjing Chen, Juan Pan, Yifu Yang, Hongwu Huang, Huiping Lai, Lei Yang, Hongyan Ai

**Affiliations:** ^1^Zhuzhou Central Hospital, Zhuzhou, 412007 Hunan, China; ^2^Department of Ultrasound, Zhuzhou Central Hospital, Zhuzhou, 412007 Hunan, China; ^3^Surgery Department, Zhuzhou Central Hospital, Zhuzhou, 412007 Hunan, China

## Abstract

Breast cancer is a highly harmful malignant tumor, which poses a great threat to women's body and mind, and the mortality rate ranks second among all women's diseases. The incidence rate accounts for 7-10% of various malignant tumors in the whole body, second only to uterine cancer in women, and has become the main cause of threatening women's health. Advanced breast cancer is often considered an incurable disease. The family of heterogeneous nuclear ribonucleoprotein complexes is composed of about 20 hnRNP proteins with molecular weights ranging from 32 to 120 kDa, and they are named according to their molecular weights. Among them, hnRNPA2 and hnRNPB1 are the two most important members of the hnRNP family, both derived from the same gene on chromosome 7p15. Therefore, research to understand the molecular mechanism and process of breast cancer progression has an important role in promoting the current medical research on breast cancer treatment methods. Therefore, studying the mechanism of tumorigenesis is the key to tumor prevention and treatment. Therefore, this paper proposes that A2/B1 promotes the stability of NRF2 mRNA and inhibits ferroptosis and cell proliferation in breast cancer cells. The article mainly introduces the disease diagnosis method based on artificial neural network and its neural network algorithm. In the experimental part, the activity of hnRNP A2/B1 on cancer cells is deeply studied. The results show that the absorbance of the MTT method increases continuously with the extension of the culture time, and the maximum reaches 1.2. This fully shows that its absorption capacity is very strong, especially after 24 hours, the absorption rate rises from 0.6 to 0.9, which shows that 24 hours is the best absorption time. And it can also be found that hnRNPA2/B1 has a significant inhibitory effect on breast cancer cells; it can reduce the effect on breast cancer cell cycle and apoptosis.

## 1. Introduction

Cancer is the number one killer in the world. Tens of thousands of people die from cancer every year. Cancer cells have the ability to proliferate, migrate, and resist apoptosis indefinitely. Recent studies have shown that the development of breast cancer and its response to treatment are associated with a large number of specific spliced oncogenes and tumor suppressors. The process of alternative splicing can produce significant misregulation in cancer, and studies have shown that it has a significant effect on the transformation of cancer cell subtypes. Among them, hnRNPA2/B1 can promote the onset of cancer, and it has been reported that hnRNPA2/B1 can promote the disease in cancers such as liver cancer and breast cancer. This paper expounds the research progress of hnRNPA2/B1 in breast cancer in recent years and comprehensively introduces its role in tumor life activities. A comprehensive understanding of the role and influence of this nuclear protein in the process of cancer disease provides a reference for further searching for therapeutic targets. The clarification of molecular signal transduction mechanism is of great significance for guiding the development of clinical drugs and related site inhibitors.

This paper mainly expounds a new neural network diagnosis method, mainly for the treatment method proposed for breast cancer, and deeply explores the role of hnRNPA2/B1 in tumor cells. The innovation of this paper is that it not only analyzes the most female breast cancer diseases at present but also proposes a disease diagnosis method based on artificial neural network, which is not only highly experimentally researchable but also interlinked. In the experimental part, not only hnRNPA2/B1 but also two control groups were studied, respectively, which also made the experimental data more accurate.

## 2. Related Work

hnRNPA2/B1 can be expressed in the cytoplasm and nucleus of normal cells, but it is not the same in different tissues and organs and different types of cells. Cancer is more and more common in real life, and the treatment of cancer is the top priority of medical work now. Dai et al. evaluated whether patients can detect autoantibodies in preclinical stage through controlled experiments and immunoassays [1]. In a recent article published in the journal, Humphries and Fitzgerald identified hnRNPA2B1 as a novel DNA-binding protein that initiates and enhances antiviral immunity, thus revealing a new aspect of DNA recognition in the nucleus [2]. Fang et al. show that several hit compounds can prevent ALS-related RNA-binding protein (RBP) TDP-43, FUS, and HNRNPA2B1-dependent RNA recruitment into SGs [3]. Tangsongcharoen et al. found two proteins, PDIA3 and ALDOA, which can prove that ZIKV infection in pregnant mothers leads to impaired infant development [4]. Although the article is aimed at analyzing hnRNPA2/B1 in each case, the article does not introduce algorithms and conduct in-depth research. Therefore, the experimental data and its conclusions are not scientific, and there are still some deficiencies.

Forecasting of meteorological data is widely used. The data obtained by Isik and Inalli from the General Administration of Meteorology is modeled by ANN and an adaptive network-based fuzzy inference system [5]. Safa et al. put ANN in agricultural production and developed an ANN model, which can predict wheat yield under different farming conditions using both direct and indirect technical methods [6]. Ascione et al. proposed a new multistage framework for cost optimization analysis via multiobjective optimization and ANN, called CASA [7]. They all conducted in-depth research on artificial neural network algorithms but did not use them in breast cancer treatment and did not study the cell activity of hnRNPA2/B1 in the process of inhibiting cancer cells [8].

## 3. ANN-Based Disease Diagnosis Method

### 3.1. Structure of ANN

ANN can basically be divided into three layers: input, implicit, and output. The essence of ANN is artificial intelligence research, that is, to use the powerful computing power of computer to simulate the information transfer process of animal neural network. The input layer corresponds to each predicted variable (similar to the stimuli received by the creature), the hidden layer corresponds to the complexity of the neural network (similar to the biological recognition and processing of stimuli), and the output layer corresponds to the target variable (similar to biological responses to stimuli). In general, when the hidden layer contains a certain number of hidden units, an ANN containing one hidden layer can be used to approximate the solution, and a 3-level ANN can solve any complex relationship. At present, it is difficult to explain it and can only be regarded as a “black box.” Cancer is by far the most complex disease the world faces, and each cancer has its own molecular signature [9]. Therefore, an in-depth understanding of the genetic alterations in each cancer is particularly important for human health [10, 11]. In theory, the cancer could be cured if the tumor cells were completely removed with surgery. Surgical resection is still the treatment of choice for early or earlier solid tumors.

#### 3.1.1. Biological Neuron Structure

In biological systems, biological neurons, also known as nerve cells, are the basic units of the nervous system. The main building blocks of nerve cells have three parts: axon, dendrite, and cell body. A schematic figure of the neuron is shown in Figure 1.

#### 3.1.2. Artificial Neuron Structure

The assumptions made by the model are as follows:

1. Neurons have threshold characteristics
2. The synaptic strength is constant
3. Synapses can be divided into inhibitory and excitatory [12, 13].
4. Each neuron is a separate information processing unit composed of one input and multiple outputs

The artificial neuron with the above characteristics is mathematically modeled [14, 15], and the mathematical model in Figure 2 is obtained, and the mathematical formulas of its input and output are as follows:

(1) $$\begin{array}{c} y=f\left(v\right)=f\left(\overset{m}{\underset{a=1}{\sum }}u_{a}x_{a}-\varphi \right). \end{array}$$

It can be seen from the above model that the actual output of the neurons in the artificial neural network is jointly determined by the input unit, the connection weight, and the threshold, and the output value can be regarded as a function of the three. In practice, the input signal *x*_*a*_(*a* = 1, 2, ⋯, *m*) often appears in the form of a vector:

(2) $$\begin{array}{c} X={\left(x_{1},x_{2},\cdots ,x_{m}\right)}^{W}\in R^{m}. \end{array}$$

The weights of the corresponding neurons are also written as weight vectors:

(3) $$\begin{array}{c} U={\left(u_{1},u_{2},\cdots ,u_{m}\right)}^{W}\in R^{m}. \end{array}$$

So, the output of a neuron in ANN is expressed as

(4) $$\begin{array}{c} y=f\left(X^{W}\cdot U-\varphi \right). \end{array}$$

#### 3.1.3. Classification of Artificial Neurons

(1) Linear neurons: its excitation function is
  (5) $$\begin{array}{c} f\left(z\right)=z \end{array}$$
(2) Threshold neuron: its excitation function is
  (6) $$\begin{array}{c} f\left(z\right)=\left\{\begin{array}{cc} 1 & z\geq 0,\\ -1 & z<0 \end{array}\right. \end{array}$$
(3) Nonlinear neurons: its sigmoid function is
  (7) $$\begin{array}{c} f\left(z\right)=\frac{1}{1+e^{-z}}, \end{array}$$
  (8) $$\begin{array}{c} \text{or }f\left(z\right)=\frac{1-e^{-z}}{1+e^{-z}} \end{array}$$

### 3.2. Classification and Topology of ANN

#### 3.2.1. Forward Network

Artificial neural networks can be divided into continuous and discrete networks, or deterministic and random networks according to their performance, and can be divided into forward networks and feedback networks according to their topology. The forward network includes single-layer perceptron, multilayer perceptron, BP, and adaptive linear neural network. The feed-forward network is also known as the feed-forward network [16], as shown in Figure 3(a).

#### 3.2.2. Feedback Forward Network

The difference between the forward feedback network and the forward network is that the specific information of the output neurons will be transmitted to the neurons of the input layer in the form of input signals, as shown in Figure 3(b) [17].

#### 3.2.3. Intralayer Interconnection Forward Network

In forward and feedback-forward networks, neurons at the same level are independent of each other, and there is no lateral connection. In a forward network with interconnected layers, neurons in the same layer can interact, as shown in Figure 4(a). This method can limit the number of neurons at each level, or divide the neurons at each level into several groups, so that each group can play a role as a whole. For example, through the lateral influence between neurons on the same level, the neuron with the highest output in this level can be selected so that other neurons cannot output [18, 19].

#### 3.2.4. Interconnection Network (Full Interconnection Network and Partial Interconnection Network)

In the Internet, two neurons in any layer can be connected to each other, as shown in Figure 4(b). In a forward network without feedback, the process is completed when a specific signal passes through a neuron [20, 21]. However, in an interconnected network, a particular piece of information can be exchanged frequently through neurons at different levels, thus making the network in a dynamic state. After many transmissions, the interconnected network will reach a kind of equilibrium [22]. However, due to the difference between the structure of the network and the properties of neurons, it is also possible to produce phenomena such as periodic oscillations and chaos.

#### 3.2.5. Learning of ANN

An instance of artificial neural network can only be used to solve various practical problems after learning and training. The strong learning ability makes artificial neural network attract the attention of various industries. Generally, ANN can be classified into two types: unsupervised learning and supervised learning, as shown in Figures 5(a) and 5(b).

### 3.3. BP Neural Network Learning Algorithm

Its network model is shown in Figure 6.

Each sample consists of a training pattern (as the input of the BP-net) and an expected pattern (as the standard output of the BP-net expected corresponding to the training pattern). Record the active value of the neuron after the input of the *z*th training mode; the input layer of the neuron has *j* neurons. Then,

(9) $$\begin{array}{c} m_{a}^{z}=\overset{m}{\underset{b=1}{\sum }}v_{ba}\cdot q_{b}^{z}, \end{array}$$

(10) $$\begin{array}{c} q_{b}^{z}=f\left(m_{a}^{z}\right)=\frac{1}{1+e^{-m_{a}^{z}}}. \end{array}$$

Define the output error of a certain layer of the BP network as follows:

(11) $$\begin{array}{c} E=\overset{i}{\underset{z=1}{\sum }}E_{z}, \end{array}$$

(12) $$\begin{array}{c} E_{z}=\frac{1}{2}\overset{j}{\underset{a=1}{\sum }}{\left(t_{a}^{z}-q_{a}^{z}\right)}^{2}, \end{array}$$

where *E* is the sum of the output errors generated by all training modes in the training set. Then, define

(13) $$\begin{array}{c} \Delta_{z}u_{ba}\propto -\frac{\partial E_{z}}{\partial u_{ba}}, \end{array}$$

since

(14) $$\begin{array}{c} \frac{\partial E_{z}}{\partial u_{ba}}=\frac{\partial E_{z}}{\partial m_{a}^{z}}\cdot \frac{\partial m_{a}^{z}}{\partial u_{ba}}. \end{array}$$

From formula (9), it can be obtained as follows:

(15) $$\begin{array}{c} \frac{\partial m_{a}^{z}}{\partial u_{ba}}=q_{b}^{z}. \end{array}$$

Reorder

(16) $$\begin{array}{c} \sigma_{a}^{z}=-\frac{\partial E_{z}}{\partial m_{a}^{z}}. \end{array}$$

Using it to represent the error correction amount, people have

(17) $$\begin{array}{c} \Delta_{z}u_{ba}={\chi \sigma }_{a}^{z}q_{b}^{z}. \end{array}$$

For output layer neurons, there are

(18) $$\begin{array}{c} \sigma_{a}^{z}=-\frac{\partial E_{z}}{\partial m_{a}^{z}}=-\frac{\partial E_{z}}{\partial a_{a}^{z}}\cdot \frac{\partial a_{l}^{z}}{\partial m_{a}^{z}}=-\left[-\left(t_{a}^{z}-q_{a}^{z}\right)\right]\cdot f^{\prime }\left(m_{a}^{z}\right)=f^{\prime }\left(m_{a}^{z}\right)\cdot \left(t_{a}^{z}-q_{a}^{z}\right). \end{array}$$

It can be ordered as follows:

(19) $$\begin{array}{c} \frac{\partial E_{z}}{\partial q_{a}^{z}}=\overset{j}{\underset{l=1}{\sum }}\frac{\partial E_{z}}{\partial m_{a}^{z}}\cdot \frac{\partial m_{l}^{z}}{\partial q_{a}^{z}}=-\overset{j}{\underset{l=1}{\sum }}\sigma_{l}^{z}v_{al}. \end{array}$$

Then,

(20) $$\begin{array}{c} \sigma_{a}^{z}=f^{\prime }\left(m_{a}^{z}\right)\cdot -\overset{j}{\underset{l=1}{\sum }}\sigma_{l}^{p}v_{al}. \end{array}$$

## 4. Deconstruction of Cancer Cell Activity by hnRNPA2/B1

### 4.1. Experimental Design

#### 4.1.1. Research Content

The breast cancers were divided into group A as the control group without transfection, group B as the negative control, and group C as the group with reduced hnRNPA2/B1 gene expression level. Green fluorescent protein was detected in the transfected cells [23]. The migration and infiltration of the cells in Transwell were measured by MTT and FCM methods, and their proliferation activity, cycle distribution, and early apoptosis were observed. The expression of p-PI3K and p-AKT mRNA in each group of rats was analyzed by fluorescence quantitative PCR technology.

#### 4.1.2. Purpose

Multiple studies have proved that hnRNPA2/B1 has a certain relationship with various diseases, but few people have explored the signaling mechanism of hnRNPA2/B1 and diseases. Therefore, understanding its molecular signaling mechanism will help guide drug development and therapy. Therefore, based on the previous work of this paper, this paper will preliminarily discuss the mechanism of hnRNPA2/B1 gene in the occurrence of breast cancer.

This study was mainly to investigate the proliferation and apoptosis of downregulated hnRNPA2/B1 gene in breast cancer cells and to explore its role in the PI3K/AKT signaling pathway, so as to determine its relationship with PI3K/AKT.

### 4.2. Deconstruction Method

#### 4.2.1. Cell Culture

*(1) Regeneration*. Separate the cell mass from the liquid nitrogen container, shake it quickly in water at about 37 degrees to dissolve all the cells in the cell quickly, centrifuge quickly with a centrifuge for 3 minutes, and absorb all the supernatant (DMSO). Add another 1 ml and stir well, then inject into a 6 mm cell culture dish, and add double antibody to prevent cell infection. After 24 hours, adherence and growth were observed. The cells were cultured in a cell culture dish at 37°C, 100% humidity, and 5% CO_2_.

*(2) Cultured Cells*. Culture various cells in DMEM contain 10% fetal bovine serum. The cells in the dish were placed in a cell culture tank with a temperature of 37°C and a humidity of 100% and were cultured in a cell culture tank containing 5% CO_2_. Monitor the cell growth every day, and change the culture medium every day or 1-2 days, and the well-grown cells can be filled in 1-2 days.

*(3) Cell Passage*. As shown in Table 1, when the cultured cells (MDA-MB-231, MCF-7) are at 80%-90%, they can be passaged. The cell condition has a great relationship with the density. Add 1 ml of 0.25% trypsin. During the digestion process, place the cell culture dish under a white light microscope with an ultraclean workbench to observe the morphology of the cells and find that the connection between the cell edges and the cells is loose, which indicates that digestion has been completed. With the rotation of the petri dish, use the tip of the long gun to suck the medium into the body. After separating all the cells, the culture solution was placed in a 4 ml sterile centrifuge tube and slowly centrifuged at 800 rpm for 3 minutes, and then, the supernatant was aspirated. The appropriate cell suspension is then poured into a new dish, followed by the addition of complete medium.

*(4) Cell Cryopreservation*. As shown in Table 2, when the fusion degree of MDA-MB-231 and MCF-7 cells is 80%-90%, the cells are cryopreserved: prepare cell cryopreservation solution in advance; prepare cryopreservation tube; the cells are in a 6 cm dish with PBS buffer 3 times; the cells were treated with 2 ml of trypsin for 1-2 minutes, followed by trypsin absorption for 1-2 minutes. Then, the trypsin was removed, 1 ml of complete culture medium was added, the cells were resuspended, and the suspension was transferred to a 1.5 ml centrifuge tube and centrifuged at a low speed of 800 rpm for 3 min in a centrifuge. Discard the supernatant, add 1 ml of freshly prepared cell cryopreservation solution, mix thoroughly and gently, and transfer the cell suspension to a sterile cryopreservation tube. Label the cryovial with the name of the cell line, the storage time, and the name of the recipient, and seal it with a sealing film. The cryovials were frozen in a 4°C refrigerator for 110 minutes, then transferred to -20°C for 20-30 minutes, then placed in -80°C for 1 day, and then placed in a liquid nitrogen container for refrigeration.

#### 4.2.2. Transfection

In the transfection method (MDA-MB-231, MCF-7), only 10% fetal bovine serum (MDA-MB-231, MCF-7) was used, and then, DNA and Lipofectamine were added to the culture medium at a ratio of 1 : 3, fully stirred to make a complex; 72 hours after transfection, a 1 mg/ml G418 culture medium was screened for 2 weeks to establish a stable transfected plasmid, which was detected under a fluorescence inversion microscope. The expression of green fluorescent protein (GFP) reflects the transfection effect of the gene. Parts of the successfully transfected cells were cryopreserved; the rest of the cells were continued to be cultured in the complete medium. After every two passages, GFP was detected by a fluorescence microscope. If the fluorescence intensity decreased, G418 continued. This study was divided into three groups: control group, negative control group, and transfection shRNA-hnRNPA2/B1 gene expression downregulation group.

#### 4.2.3. Determination of Cell Cycle and Apoptosis by FCM Method

Take 1 × 10^6^ mice, add 70% ice alcohol solution, and let it stand at 4°C. In the next day, the ice alcohol was removed by centrifugation, PI and RNase A were added, and after 30 minutes, the cells were washed three times with PBS, and then, the ratio of G1, S, and G2 was measured by an upper flow cytometer produced by BD Company in the United States. Take 5 × 10^5^ cells of each group, resuspend them in 500 ml PBS, add 2 ml Annexin V-psycoerythrocytes (PE) and mix them with 10 ml 7-ADD, and incubate for 15 minutes, rinse with PBS, and then measure the apoptosis rate by flow cytometry. The test was performed 5 times.

Statistical data were carried out using SPSS21.0 software, and statistical data expressed by *x* ± *s* were compared by group using one-way variance, and *P* < 0.05 indicated a significant difference.

### 4.3. Main Technology

1. At a concentration of 3 ng/nl (the protein concentration is diluted with RIPA dissolution solution), 5x loading buffer and protein sample are mixed at a volume of 1 : 4. Protein denaturation was then performed in PCR at 100°C for 5 minutes
2. Select the appropriate separation gel concentration according to the protein size, coat a layer of double-distilled water sealant on the surface of the colloid, and let it stand for 1 hour at room temperature. After the release glue has cured, let the double vapor out; add the 5% strength adhesive, fill it with the remaining glass pieces (about 4 ml/piece), and insert the comb into the concentrated glue to prevent air bubbles. After 30 minutes at room temperature, put the prepared glass pieces in a 200 ml electric pool, soak for 1-2 minutes, and then gently pull out with a brush. Add 30 l of protein sample (90 g in total) to the sample well, use a small well as a marker well, and add 5 *μ*l of protein marker. Make up to 30 *μ*l with RIPA dissolution solution and 5x loading buffer at a volume ratio of 4 : 1 to ensure the same number of injections per well. Stacking gel constant pressure 70 V, 60 minutes, 100 V, 150 minutes, glue constant pressure
3. After the electrophoresis is completed, the target strip is cut according to the Martens strip, and then, the filter paper with the appropriate size and the size of the strip is combined with the PVDF film. Immerse the PVDF film for 15 seconds and place it in 1x transfer buffer; soak the transfer device (clip, filter, and filter paper) with precooled 1x transfer buffer, and then, assemble the clamp into a clip. Sponge PVDF membrane and other tools are placed in order to discharge air bubbles, so that glue, filter paper, and PVDF membrane can be accurately bonded. The transfer sheet is placed in the transfer trough and filled with precooled spinning film buffer. Place the entire device in the refrigerator on a rotating film kept at low temperature. A constant current of 200 mA was used for the film for 50 minutes; the protein-coated PVDF film was placed in TBST buffer and washed 3 times for 5 minutes
4. Remove the PVDF film from the TBST buffer, inject 5% skim milk (0.01 MTBST dilution) into the antibody incubator, block at room temperature, and shake for 2-3 hours to eliminate the nonspecific binding of the antibody. Discard blocking solution; add 3 ml of antiflush, overnight at 4°C; perform 5 TBST washes, 5 min each at room temperature. Incubate 3 ml of HRP-conjugated secondary antibody for 2 hours at room temperature; wash 5 times with TBST for 5 minutes each
5. Mix 1 ml each of ECL reagent A and B solutions, and contact the working liquid with the protein side of the PVDF film downward. After 3 minutes, the residual fluorescent liquid was blotted dry with filter paper, and then, the protein of the PVDF film was put into the dark box, then transferred to the dark room, exposed in the dark box, and then rinsed and fixed in sequence
6. Real-time quantitative PCR RNA method: (1) take out even-numbered growth phase cells, absorb the old medium, and add PBS to wash 3 times. (2) Add 1 ml of TRIzol for 5 minutes, during which time the cell lysis is made easier by blowing air. (3) Add 1 ml of thermal lysis solution to 200 ml of chloroform, mix up and down 15 times, and let it stand for 5 minutes. (4) Centrifuge at 4°C, 12,000 rpm for 15 minutes. (5) Divide the solution obtained after centrifugation into three layers, the top layer of which is the desired RNA, and then, pipette it into an EP tube without RNase. (6) RNA precipitation: add precooled isopropanol, turn it upside down, and stir repeatedly. (7) RNA washing: remove the supernatant prepared with DEPC water, and rinse the coated RNA pellet with alcohol once. Centrifuge at 7500 rpm for 5 minutes at 4°C. (8) Redissolution of RNA: place 10 min at room temperature to evaporate hexanol. Add a proportion of DEPC water to dissolve it. (9) Concentration meter purity test: mix 1 ml of RNA with 99 ml of DEPC water to test its purity and content
7. The reverse transcription reaction occurs based on the RNA concentration
8. miRNA reverse transcription: turn the reagents (RNA solution, RNase-free double-distilled water, and buffer) required for miRNA reverse transcriptase upside down, mix well, and then temporarily put it into ice for use. Use 25 *μ*l miRNA reverse transcription system in RNase-free EP tubes, after brief separation, 37°C, 60 minutes, 85°C, 5 minutes. The reverse transcriptase was diluted 5 times with sterile water
9. miRNA real-time quantitative PCR: dilute the universal adaptor PCR primer to 2 *μ*l with RNase-free double steam water. Prepare 20 *μ*l of qPCR reaction solution on ice, mix the reaction solution well, then add it to the PCR reactor, and perform a brief centrifugation to ensure the bottom of the reaction tube, one cycle for 10 minutes at 95°C, one cycle for 20 minutes at 58°C, and one cycle for 10 minutes at 72°C, 30 cycles. The target gene and the reference gene were subjected to quantitative PCR to obtain the CT value, and the relative expression of each sample gene was compared by 2-△CT technology. The gene expression level of each group was set to 1, and the related expression levels of the other two groups were calculated and plotted according to the correlation fold. According to the results of the experimental control group, 2-CT showed the fold variation of target gene expression in the experimental group

### 4.4. Results and Deconstruction

1. Detection of cell viability by MTT method: collect cells from the control group, negative control group, and hnRNPA2/B1 downregulation group, and inoculate 5000 cells/well in 96-well plates, respectively. After culturing for 6, 12, 24, 48, 72, and 96 h, add 20 ml of MTT solution to each well for 4 h, then discard the supernatant, and add 150 ml of DMSO for slight shaking for 5 min. Then, the absorbance (D) value of each group was detected at a wavelength of 492 nm to reflect the proliferation activity of each group of cells. The experiment was repeated 5 times. The results are shown in Figure 7

According to the results, the absorbance (D) value of the MTT method for cell viability detection data will continue to increase with the continuous growth of the culture time, until it reaches 1.2, which is enough to indicate that its activity absorption rate is very good, especially at 24 hours. After that, it increased from 0.6 directly to the absorption rate of 0.9, which also indicated that 24 hours was the best time.

(2) Transwell cell migration and infiltration test: 12 hours after the start of the test, the basement membrane was hydrated with 50 ml of serum-free medium after drying with Matrigel at 37°C for 25 minutes, and the cell migration test was carried out. First, perform conventional centrifugation, wash twice, adjust the concentration of cells to 1 × 10^4^/ml, and inject 200 ml of cell suspension into the chamber and 500 ml of fetal bovine serum in the lower chamber. The 24-hour culture chamber was taken out, rinsed with PBS, and wiped. After 6 minutes, soak in alcohol for 6 minutes, and then, use it for 15 minutes, randomly select 10 fields of view, and calculate the average value of transmembrane cells.  Figure 8 shows the cell migration and infiltration assay (Figure 8(a) represents cell migration; Figure 8(b) represents cell infiltration; *P* < 0.001).
(3) The expression of hnRNPA2/B1, p-PI3K, and p-AKT mRNA in each group of cells was detected by real-time fluorescence quantitative PCR, as shown in Table 3
(4) Detection of p-PI3K and p-AKT protein expressions in the cells of each group by western blot, as shown in Table 4
(5) Detection by MTT method and FCM method

According to the test data of MTT method and FCM method for each group of cells, it can be seen that the effect of MTT method is better than that of FCM method (Figures 9(a) and 9(b)).

To sum up, experiments to clarify the operation mechanism of breast cancer from the onset to the deterioration are particularly important for the identification of its potential molecular therapeutic targets and breast cancer treatment research. The development of breast cancer and its response to treatment are associated with a number of specific spliced oncogenes and tumor suppressors. The process of alternative splicing can produce significant misregulation in cancer, and studies have shown that it has a significant effect on the transformation of cancer cell subtypes.

## 5. Conclusions

According to the research of A2/B1 promoting the stability of NRF2 mRNA and inhibiting ferroptosis and cell proliferation in breast cancer cells, the results can show that knockdown of hnRNPA2/B1 can reduce the viability of breast cancer cells, change the cell cycle of breast cancer, and increase cell apoptosis. Knockdown of hnRNPA2/B1 can reduce the proliferation and invasion of breast cancer cells, reduce the expression of PI3K/AKT signaling-related protein and mRNA, and inhibit its activation. Some spliceosome-mutated elements are also predicted to lead to driver mutations in many cancers, providing strong evidence for the important role of splicing factors in cancer development. However, little is known about the specific roles of splicing factors in the occurrence and development of cancer. By upregulating the mRNA level of hnRNPA2/B1 to increase its protein expression, the cell proliferation ability, tumorigenic ability, and cell biological activity were improved. In this study, people analyzed the inhibitory effect of knockdown of hnRNPA2/B1 on the invasion and proliferation of breast cancer cells through PI3K/AKT signaling and provided a laboratory basis for targeted therapy of clinical patients.

## Figures and Tables

**Figure 1:** Schematic figure of biological neuron structure.

**Figure 2:** Schematic figure of the M-P model.

**Figure 3:** ANN network classification figure.

**Figure 4:** Schematic figure of intralayer interconnection forward network and interconnection network.

**Figure 5:** ANN learning figure.

**Figure 6:** Schematic figure of BP neural network model.

**Figure 7:** Detection of cell viability by MTT assay.

**Figure 8:** Cell migration and invasion assays.

**Figure 9:** Test data of each group of cells by MTT method and FCM method.

**Table 1:** Confluence of three groups of cultured cells.

	MDA-MB-231	MCF-7
Group A	89%	82%
Group B	84%	87%
Group C	81%	90%

**Table 2:** Confluence of three groups of cultured cells after cryopreservation.

	MDA-MB-231	MCF-7
Group A	74%	62%
Group B	64%	77%
Group C	61%	81%

**Table 3:** Three groups of PCR detection of protein expression.

	hnRNPA2/B1	p-PI3K	p-AKT mRNA
Group A	1.17 ± 0.06	0.58 ± 0.12	1.37 ± 0.34
Group B	1.23 ± 0.11	0.89 ± 0.14	2.31 ± 0.19
Group C	1.56 ± 0.13	1.10 ± 0.23	3.19 ± 0.31
*F*	14.221	11.071	18.234
*P*	<0.001	<0.001	<0.001

**Table 4:** Expression of p-PI3K and p-AKT proteins in the cells of each group.

Group	p-PI3K protein expression	p-AKT protein expression
Group A	1.29 ± 0.16^a^	0.89 ± 0.12^a^
Group B	1.23 ± 0.17^a^	0.85 ± 0.13^a^
Group C	0.82 ± 0.14	0.60 ± 0.09
*F*	16.372	14.290
*P*	<0.001	<0.001

## Data Availability

The data that support the findings of this study are available from the corresponding author upon reasonable request.

## References

[1] Dai L., Li J., Tsay J., Xiao W., Zhang J. Y. (2017). Abstract 710: identification of autoantibody to ECH1 & HNRNPA2B1 as potential biomarkers in the early detection of lung cancer. *Cancer Research*.

[2] Humphries F., Fitzgerald K. A. (2019). hnRNPA2B1: fueling antiviral immunity from the nucleus. *Molecular Cell*.

[3] Fang M. Y., Markmiller S., Vu A. Q. (2019). Small-molecule modulation of TDP-43 recruitment to stress granules prevents persistent TDP-43 accumulation in ALS/FTD. *Neuron*.

[4] Tangsongcharoen C., Roytrakul S., Smith D. R. (2019). Analysis of cellular proteome changes in response to ZIKV NS2B-NS3 protease expression. *Biochimica et Biophysica Acta (BBA) - Proteins & Proteomics*.

[5] Isik E., Inalli M. (2018). Artificial neural networks and adaptive neuro-fuzzy inference systems approaches to forecast the meteorological data for HVAC: the case of cities for Turkey. *Energy*.

[6] Safa M., Samarasinghe S., Nejat M. (2018). Prediction of wheat production using artificial neural networks and investigating indirect factors affecting it: case study in Canterbury province, New Zealand. *Journal of Agricultural Science & Technology*.

[7] Ascione F., Bianco N., De Stasio C., Claudio M. G. M., Vanoli G. P. (2017). CASA, cost-optimal analysis by multi-objective optimisation and artificial neural networks: a new framework for the robust assessment of cost-optimal energy retrofit, feasible for any building. *Energy & Buildings*.

[8] Arslan E., Koyuncu I. (2021). Comparison of amino acid metabolisms in normal prostate (PNT-1A) and cancer cells (PC-3). *Oncologie*.

[9] Ahmed N., Masri A., Mokayed H. (2020). An efficient machine learning based cervical cancer detection and classification. *Journal of Cybersecurity and Information Management*.

[10] Cascardi A., Micelli F., Aiello M. A. (2017). An artificial neural networks model for the prediction of the compressive strength of FRP-confined concrete circular columns. *Engineering Structures*.

[11] Ascione F., Bianco N., Stasio C. D., Mauro G. M., Vanoli G. P. (2017). Artificial neural networks to predict energy performance and retrofit scenarios for any member of a building category: a novel approach. *Energy*.

[12] Mansourian S., Darbandi E. I., Mohassel M. R., Rastgoo M., Kanouni H. (2017). Comparison of artificial neural networks and logistic regression as potential methods for predicting weed populations on dryland chickpea and winter wheat fields of Kurdistan province Iran. *Crop Protection*.

[13] Cervone G., Clemente-Harding L., Alessandrini S., Delle Monache L. (2017). Short-term photovoltaic power forecasting using Artificial Neural Networks and an Analog Ensemble. *Renewable Energy*.

[14] Bazan G. H., Scalassara P. R., Endo W. (2017). Stator fault analysis of three-phase induction motors using information measures and artificial neural networks. *Electric Power Systems Research*.

[15] García-Segura T., Yepes V., Frangopol D. M. (2017). Multi-objective design of post-tensioned concrete road bridges using artificial neural networks. *Structural and Multidisciplinary Optimization*.

[16] Giovanis D. G., Papaioannou I., Straub D., Papadopoulos V. (2017). Bayesian updating with subset simulation using artificial neural networks. *Computer Methods in Applied Mechanics & Engineering*.

[17] Nejad F. P., Jaksa M. B. (2017). Load-settlement behavior modeling of single piles using artificial neural networks and CPT data. *Computers and Geotechnics*.

[18] Mahbod A., Chowdhury M., Smedby O., Orjan C. W. (2018). Automatic brain segmentation using artificial neural networks with shape context. *Pattern Recognition Letters*.

[19] Sitton J. D., Zeinali Y., Story B. A. (2017). Rapid soil classification using artificial neural networks for use in constructing compressed earth blocks. *Construction and Building Materials*.

[20] Paradarami T. K., Bastian N. D., Wightman J. L. (2017). A hybrid recommender system using artificial neural networks. *Expert Systems with Applications*.

[21] Morfidis K., Kostinakis K. (2018). Approaches to the rapid seismic damage prediction of r/c buildings using artificial neural networks. *Engineering Structures*.

[22] Kocadagli O., Langari R. (2017). Classification of EEG signals for epileptic seizures using hybrid artificial neural networks based wavelet transforms and fuzzy relations. *Expert Systems with Applications*.

[23] Li X., Wang Y., Zhao Y., Wei Y. (2022). Fast speckle noise suppression algorithm in breast ultrasound image using three-dimensional deep learning. *Frontiers in Physiology*.

